# A Cohort Study to Compare Effects between Ulcer- and Nonulcer-Related Nonvariceal Upper Gastrointestinal Bleeding

**DOI:** 10.1155/2022/3342919

**Published:** 2022-06-10

**Authors:** Bi Nian, Bangping Wang, Long Wang, Lanjuan Yi

**Affiliations:** ^1^Department of Gastroenterology, Suzhou First People's Hospital, China; ^2^Gastroenterology Department, Suzhou Municipal Hospital, China; ^3^Department of Gastroenterology, Yantai Mountain Hospital, Yantai, China

## Abstract

**Objective:**

The aim of this study was to better understand the characteristics and etiology of acute nonvariceal upper gastrointestinal bleeding (ANVUGIB) in recent years in this region and to provide evidence-based medical evidence.

**Methods:**

100 patients with acute nonvariceal upper gastrointestinal bleeding (ANVUGIB) who met the clinical diagnostic criteria of ANVUGIB admitted to Suzhou First People's Hospital from January 2017 to December 2021 were analyzed, as well as the age difference and change rule. According to age, 100 patients were divided into young (18-39 years), middle-aged (40-59 years), and elderly (60 years and above), and the differences in the three groups were compared. The etiology was confirmed by endoscopic examination and was recorded one by one in a well-designed ANVUGIB case data registration form. Statistical software SPSS 23.0 was used for analysis.

**Results:**

Gastric ulcer was the main cause in the elderly group (50.0%), duodenal ulcer was the main cause in the middle and young groups, and gastrointestinal cancer (7.1%) and marginal ulcer (2.3%) in the elderly group were higher than those in the young group. Nonsteroidal anti-inflammatory drugs (52.3%) were the main inducement in the elderly group, which was significantly higher than in the middle-aged group (13.1%) and the young group (5%) (*P* < 0.01). Drinking, fatigue, and emotional excitement led to a higher proportion in the middle-aged group and the young group, in comparison to the elderly group (*P* < 0.01).

**Conclusion:**

Peptic ulcer is the most common cause of acute nonvariceal upper gastrointestinal bleeding, followed by acute gastric mucosal lesions and upper digestive system tumors, compared with nonulcer.

## 1. Introduction

Acute nonvariceal upper gastrointestinal bleeding (ANVUGIB) refers to bleeding caused by nonvariceal diseases of the digestive tract above the flexion ligament, including bleeding from the pancreas and biliary tract and bleeding caused by diseases near the anastomosis after gastrojejunostomy, with an annual incidence of 50~150/100,000, and a case fatality rate of 6%~10% [1]. It is a common acute and critical disease of the digestive system, with rapid onset, rapid progress, dangerous condition, and high fatality rate [2]. Therefore, the diagnosis and treatment of ANVUGIB is still a hot spot in clinical research at home and abroad [3]. Includes statistical analysis of the etiological composition, changing patterns, timing and endoscopic treatment methods of ANVUGIB in the region. In order to better understand the etiological characteristics and changes of ANVUGIB in recent years, we must deepen the understanding of ANVUGIB by clinicians and provide evidence-based medical evidence to guide clinical treatment [4–6]. With the continuous popularization and development of endoscopic technology since the late 1990s, great progress has been made in the etiological diagnosis and treatment of ANVUGIB, which gives us a preliminary understanding of the etiological composition of ANVUGIB [7]. However, in the past 10 years, As we learn more about H. pylori, more standardised strategies for H. pylori eradication are becoming more common [8]. As a result, the incidence of HP-related digestive ulcer bleeding continues to decrease. At the same time, the aging of China's population is increasingly aggravated, and the incidence of serious basic diseases such as cardiovascular and cerebrovascular diseases is increasing year by year. Nonsteroidal anti-inflammatory drugs (NSAIDs) are a major treatment for cases of upper gastrointestinal hemorrhage [9, 10]. However, NSAIDs also have many side effects, most commonly in the gastrointestinal tract, cardiovascular system, kidney, liver, and central nervous system as well as the hematopoietic system [11]. Endoscopic therapy plays an increasingly important role in the treatment of ANVUGIB. The comparison of different endoscopic treatment methods and the best choice of endoscopic treatment timing can not only greatly improve the cure rate but also save medical resources, so that patients can obtain the maximum benefit.

Therefore, the clinical characteristics of ANVUGIB, such as inducing factors, etiology composition, and onset age, have undergone corresponding changes [12]. It is of great significance to seriously summarize the characteristics and incidence rules of ANVUGIB for guiding clinical work, improving cure rate, and reducing mortality [13]. Due to differences in the medical environment, economic status, disease spectrum and lifestyles in different regions, the etiological composition of acute nonvariceal upper gastrointestinal bleeding is also different [14]. Up to now, there is still a lack of relevant large-sample investigations in Anhui Province and even Southeast China on the change rule of the etiological composition of acute nonvariceal upper gastrointestinal bleeding [15, 16].

With the continuous development and improvement of endoscopic treatment technology, the advantages of endoscopic treatment for acute nonvariceal upper gastrointestinal bleeding are becoming more and more obvious, which greatly reduces the mortality, rebleeding rate, and surgical treatment rate of bleeding patients, saves resources and reduces costs, and opens a new chapter for the treatment of ANVUGIB [17–19]. Therefore, the understanding of the etiological composition and the change of factors such as inducement is of great importance to guide treatment and improve prognosis [20].

This study will carry out a large-sample clinical epidemiological study to clarify the etiological structure, variation, and influencing factors of acute nonvariceal upper gastrointestinal bleeding, in order to clarify the etiology for improving prognosis and guiding treatment.

## 2. Materials and Methods

### 2.1. Object of Study

Medical records of a total of 100 inpatients who met the clinical diagnostic criteria of ANVUGIB and had the etiology confirmed by endoscopic examination from January 2017 to December 2021 were included. According to age, the 100 patients were divided into young (18-39 years), middle-aged (40-59 years), and elderly (60 years and above), and the differences in the three groups were compared. Age ranged from 18 to 96 years, with an average of 54.6 ± 16.3 years. There were 80 males and 20 females, with a male to female ratio of about 4:1.

### 2.2. Inclusion Criteria

(1) The patient presents symptoms of hematemesis and/or melena, which may be accompanied by dizziness, pallor, increased heart rate, decreased blood pressure, and other signs of peripheral circulatory failure, and the diagnosis of acute upper gastrointestinal bleeding is established. (2) Endoscopic examination found nonvariceal bleeding lesions in the upper digestive tract, and ANVUGIB diagnosis could be established.

### 2.3. Exclusion Criteria

(1) We exclude patients with bleeding from lesions of the mouth, nose, pharynx, or respiratory tract. (2) We exclude patients who are taking some drugs (such as iron and bismuth) and food (such as animal blood) or have black stool. For suspicious patients, gastric juice, vomit, or fecal occult blood test can be performed. (3) Lower gastrointestinal bleeding and bleeding caused by esophagogastric varices were excluded. (4) Patients younger than 18 years old and without endoscopic examination to determine the cause of bleeding were excluded.

### 2.4. Efficacy Evaluation Criteria

(1)*Calibration criteria for successful hemostasis*: after treatment, the bleeding was stopped under gastroscopy, the patient's condition was stable, vital signs were stable, there were no signs of active bleeding and no hematemesis and large amounts of melena, the stool gradually turned yellow, and stool specimens was negative. [2] *Criteria for rebleeding*: one of the following conditions occurs after the first successful hemostasis treatment: hematemesis, melena/hematochezia, the stomach tube sucks out fresh blood, hemodynamic instability (systolic blood pressure < 100 mmHg, heart rate > 100 beats/min, hemoglobin decrease > 20 g/L), and rebleeding was confirmed under endoscopy. [3] *Criteria for the effectiveness of endoscopic treatment*: the first endoscopic treatment was successful and there was no further bleeding within 3 days (Table 1).

### 2.5. Design Scheme

The design scheme is as follows: well-designed ANVUGIB case data registration form was signed, recording The general data of 100 ANVUGIB patients (including name, gender, and age) and date of visit were recorded by details; while also contained inducement before onset and Rockall score; and treatment method, endoscopic time, endoscopic diagnosis, Forrest grade, and disease outcome of patients (whether endoscopic treatment is effective, death, and rebleeding, etc.).

### 2.6. Statistical Analysis

Continuous data are expressed as the means ± SDs. All statistical calculations were carried out using SPSS 23.0 software. A chi-square test was used to compare count data and groups. For multiple comparisons, data were analyzed via analysis of variance (ANOVA) with the Tukey-Kramer Multiple Comparison Test. *P* values < 0.05 were considered significant.

## 3. Result

### 3.1. General Clinical Characteristics of the Patients

There were 100 patients, 80 men and 20 women, with a male to female ratio of approximately 4 : 1. Age 18~96 years, with a mean of 54.6 ± 16.3 years, included 42 elderly patients aged 60 years, 38 middle-aged patients aged 40~59 years, and 20 young patients aged 18-39 years.

### 3.2. Treatment and Outcome

After admission, all patients were given symptomatic treatment such as fasting, fluid rehydration, and acid preparation. For patients with serious conditions and hemodynamic changes, supportive treatments such as dilatation, blood transfusion, and correction of shock should be performed to maintain blood pressure stability and correct hemoglobin to more than 70 g/L. An endoscopic examination was performed as soon as possible, and an electronic gastroscope was used for the operation. ECG monitoring and high flow oxygen inhalation (oxygen flow 4-5 L/min) were performed during the examination. The etiology was confirmed by endoscopic diagnosis, and endoscopic treatment was performed according to the needs of the disease. Among the 100 patients, 2 cases had rebleeding after admission. None of the patients died in the hospital because seriously ill patients were discharged automatically,. And 2 gastric cancer bleeding cases were transferred to surgical treatment. The 100 patients were followed up by telephone after discharge, and 2 patients had died, both of them died from non bleeding-related diseases, including 1 patient with advanced tumor consumption, and 1 patient with cardiovascular and cerebrovascular diseases.

### 3.3. Comparison of Etiology in Different Age Groups

The results showed that peptic ulcer was mainly used in the three groups, with ulcer disease in the old group reaching 76.1% and 88.8% in the young group. Ulcer disease accounted for 86.8% of the middle-aged group (Table 2).

### 3.4. Comparison of Triggers for Different Age Groups

The main causes of the elderly group were nonsteroidal drugs (52.3%), which was significantly higher than in the middle-aged group (13.1%) and young group (5%), *P* < 0.01, and for the middle and others, the main causes were drinking and fatigue, which was significantly higher than for the elderly group (*P* < 0.01). Overall, there were no significant differences between NSAIDs, drinking, and exertion among the three major triggers (*P* > 0.05). ALL patients were common in acute nonvariceal upper gastrointestinal bleeding predisposition (Table 3).

### 3.5. Difference in Effective Rate with Different Forrest Grades

Analyzing the treatment efficiency of different treatment groups with different Forrest grades, we show that, overall, grade Forrest II lesions are more efficient than each treatment method of grade Forrest lesions. For grade Forrest Ia and A lesions, titanium clamp and combination treatment were highly efficient, significantly higher than in the injection and APC electrocoagulation groups (*P* < 0.05, statistically significant difference). In the combined treatment group, 91.3% of grade IA and grade IIA lesions were treated by titanium clip combined with submucosal epinephrine injection. Therefore, mechanical clamping of the titanium clip is the main treatment method for grade IA lesions and grade IIA lesions, and the immunohistochemistry of gastrointestinal bleeding tissue is shown in Figure 1.

## 4. Discussion

ANVUGIB is mainly caused by diseases of the upper digestive tract and biliary and pancreatic diseases. Peptic ulcers, upper gastrointestinal tumor, and acute gastric mucosal lesions were the most common [21]. This study showed that the most common causes of acute nonvaricose upper gastrointestinal bleeding were peptic ulcer, acute gastric mucosal lesion, and upper gastrointestinal tumor, and other causes were esophagocardiac mucosal tear syndrome [22]. The etiological distribution is similar to that reported in related studies. In this study, peptic ulcer is still the main cause of bleeding, accounting for 81%, especially duodenal ulcers, which is consistent with the incidence reported in the past [23–26]. The difference between the two groups was statistically significant, which was consistent with literature reports [27]. Gastric ulcers are relatively more common in elderly patients due to decreased secretion of gastric acid and pepsin and decreased defence ability due to gland atrophy, while duodenal ulcers due to high acid secretion are relatively less common. In addition, the elderly often need to take a large number of NSAIDs for a long time, and the incidence of gastric ulcers associated with NSAIDs is increasing, which is often characterized by multiple ulcers. In gastric erosive bleeding, the lesion is in the fundus, followed by the horn and sinus. With age, the blood flow to the gastric mucosa decreases, and the synthesis and secretion of mucus and carbonate decrease, both leading to a gradual decrease in the defensive function of the gastric mucosa. When the mucosa is stimulated by NSAIDs, prostaglandin synthesis decreases, further reducing the defences of the mucosa; at the same time, the increase in reverse diffusion of hydrogen ions aggravates the damage to the mucosa and directly causes bleeding [28, 29]. In addition, NSAIDs can inhibit thromboxane synthesis, reduce platelet aggregation, inhibit nitric oxide synthase (cNOS), reduce the synthesis of NO that can protect gastrointestinal mucosa, and induce the increase of the inflammatory mediator leukotriene (LT), thus aggravating mucosal damage and inducing bleeding [30].

In addition to ulcer disease, the upper gastrointestinal tumor was the second cause of acute nonvariceal upper gastrointestinal bleeding [31]. Due to canceration of ulcers and decreased immune function, upper gastrointestinal tumors are more frequent in elderly patients, thus accounting for a higher proportion of acute nonvariceal upper gastrointestinal bleeding than in young and middle-aged groups [32]. For acute nonvariceal upper gastrointestinal bleeding in the elderly, we should be vigilant with gastric cancer bleeding and pay attention to its identification, and repeated gastroscopy and biopsy can improve the positive rate of diagnosis, so as not to delay the best time for diagnosis and treatment [33, 34]. With the development and popularization of endoscopic technology, the immediate hemostasis rate of endoscopic hemostasis can be as high as nearly 100%, which significantly reduces the surgical emergency operation rate, rebleeding rate, and total mortality rate [35]. Therefore, emergency endoscopy has become the preferred method for the diagnosis and treatment of acute upper gastrointestinal bleeding [36].

The advantage of this study was to demonstrate the importance of ulcer in the progress of nonvariceal upper gastrointestinal bleeding, which was brought to light for the future prevention and treatment of this disease. However, there are also limits to this study. First, the number of patients is not so large, which needs further validation in future. Second, the mechanism was not clarified. Further studies are needed to carry more experiments to explain it.

## 5. Conclusion

Peptic ulcer is the most common cause of acute nonvariceal upper gastrointestinal bleeding, followed by acute gastric mucosal lesions and upper digestive system tumors, compared with nonulcers. Among the causes of acute nonvariceal upper gastrointestinal bleeding, gastric ulcers were mainly found in the elderly group, while duodenal ulcers in the middle and young groups, and the proportion of tumors in the elderly group was higher than that in the younger group.

## Figures and Tables

**Figure 1:** Immunohistochemistry of human upper gastrointestinal ulcer tissue (histological staining and immunohistochemical staining of IgE).

**Table 1:** Forrest grading of peptic ulcer.

Forrest grading	Ulcer lesions	Probability of rebleeding
Ia	Jet bleeding	55%
Ib	Active oozing	55%
IIa	Blood vessels exposed	43%
IIb	Blood clot	22%
II c	Bottom of the black	10%
III	Bottom of the clean	5%

**Table 2:** Etiological composition in different age groups.

Groups	Young group	Middle-aged group	Middle-aged group	Total
*N*	20	38	42	100
Mallord-Weiss Syndrome	1	1	1	3
Reflux esophagitis	1	1	3	5
Gastric ulcer	1	9	21	31
Duodenal ulcer	15	23	10	48
Marginal ulcer	0	1	1	2
Acute gastric mucosal lesions	2	2	3	7
Esophageal cancer and Gastric cancer	0	1	3	4

**Table 3:** The composition of triggers in different age groups.

Groups	Young group	Middle-aged group	Middle-aged group	Total
Nonsteroidal anti-inflammatory drugs	1	5	22	28
Drink	12	13	3	28
Tired mood excited	5	13	10	28
Unknown cause	2	7	7	16

## Data Availability

The data used to support this study are available from the first author upon request.
